# Carnosol Attenuates LPS-Induced Inflammation of Cardiomyoblasts by Inhibiting NF-*κ*B: A Mechanistic *in Vitro* and *in Silico* Study

This article has been retracted.

**DOI:** 10.1155/2022/7969422

**Published:** 2022-05-04

**Authors:** Vafa Baradaran Rahimi, Mohammad Amin Momeni-Moghaddam, Maria Giovanna Chini, Anella Saviano, Francesco Maione, Giuseppe Bifulco, Pouria Rahmanian-Devin, Ali Jebalbarezy, Vahid Reza Askari

**Affiliations:** ^1^Department of Cardiovascular Diseases, Faculty of Medicine, Mashhad University of Medical Sciences, Mashhad, Iran; ^2^Department of Nutrition and Biochemistry, Gonabad University of Medical Sciences, Gonabad, Iran; ^3^Department of Biosciences and Territory, University of Molise, Contrada Fonte Lappone, Pesche, Isernia I-86090, Italy; ^4^Immuno Pharma Lab, Department of Pharmacy, School of Medicine and Surgery, University of Naples Federico II, Naples, Italy; ^5^Department of Pharmacy, University of Salerno, Via Giovanni Paolo II 132, Fisciano, Salerno 84084, Italy; ^6^Department of Pharmaceutical Sciences in Persian Medicine, School of Persian and Complementary Medicine, Mashhad University of Medical Sciences, Mashhad, Iran; ^7^Department of Persian Medicine, School of Persian and Complementary Medicine, Mashhad University of Medical Sciences, Mashhad, Iran; ^8^Applied Biomedical Research Center, Mashhad University of Medical Sciences, Mashhad, Iran

## Abstract

Carnosol possesses several beneficial pharmacological properties. However, its role in lipopolysaccharide (LPS) induced inflammation and cardiomyocyte cell line (H9C2) has never been investigated. Therefore, the effect of carnosol and an NF-*κ*B inhibitor BAY 11-7082 was examined, and the underlying role of the NF-*κ*B-dependent inflammatory pathway was analyzed as the target enzyme. Cell viability, inflammatory cytokines levels (tumor necrosis factor-*α* (TNF-*α*), interleukin (IL)-1*β*, IL-6, and prostaglandin *E*_2_ (PGE_2_)), and related gene expression (TNF-*α*, IL-1*β*, IL-6, and cyclooxygenase-2 (COX-2)) were analyzed by ELISA and real-time PCR. In addition, docking studies analyzed carnosol's molecular interactions and binding modes to NF-*κ*B and IKK. We report that LPS caused the reduction of cell viability while enhancing both cytokines protein and mRNA levels (*P* < 0.001, for all cases). However, the BAY 11-7082 pretreatment of the cells and carnosol increased cell viability and reduced cytokine protein and mRNA levels (*P* < 0.001 vs. LPS, for all cases). Furthermore, our *in silico* analyses also supported the modulation of NF-*κ*B and IKK by carnosol. This evidence highlights the defensive effects of carnosol against sepsis-induced myocardial dysfunction and, contextually, paved the rationale for the next *in vitro* and *in vivo* studies aimed to precisely describe its mechanism(s) of action.

## 1. Introduction

The inflammatory response is considered one of the body's defence mechanisms as opposed to infections, chemical exposure, and injuries, which are magnified by the innate immune system's receptors. In this regard, some of the receptors detect noxious agents, leading to a specific inflammatory response by producing and secreting cytokines [1–4]. Moreover, the uncontrolled inflammatory response may result in many diseases, including cardiovascular dysfunctions, autoimmune, allergies, and cancer diseases [1, 5].

Sepsis refers to the systemic inflammatory response of the body to infections, which leads to myocardial depression and multiorgan dysfunction [5–8]. Lipopolysaccharide (LPS), a component of the Gram-negative bacteria's outer membrane, leads to septic cardiac dysfunction, causing death in patients [2, 5, 9]. Besides, LPS interacts with the cell surface toll-like receptor 4 (TLR-4) and stimulates an intracellular cascade for activating nuclear factor-kappa B (NF-*κ*B) [5, 10, 11]. Meanwhile, NF-*κ*B controls various genes involved in the inflammation process and regulates related factors, including cyclooxygenase-2 (COX-2), proinflammatory cytokines (such as interleukin (IL)-1*β*, IL-6, and tumor necrosis factor (TNF)-*α*), and vascular endothelial growth factor (VEGF) [12, 13].

Nowadays, several studies are performed to find new and effective medications for inflammatory diseases due to the increasing prevalence worldwide [14]. Several investigations demonstrated that phytochemicals have various modulatory effects on the inflammatory pathways by regulating gene expression or interaction with specific receptors and signaling pathways [15]. A representative example comes from Rosemary (*Rosmarinus officinalis*), a *Lamiaceae* family member, including lots of phytochemicals such as medioresinol, p-coumaric acid, rosmarinic acid, luteolin, apigenin, carnosic acid, and carnosol. Most anti-inflammatory properties seem to be related to carnosol and carnosic acid, which act as modulators of the arachidonic acid cascade [16–18].

Carnosol is a bioactive ortho-diphenolic diterpene associated with the abietane carbon skeleton. It has been shown that Rosemary (*R. officinalis*) and Sage (*Salvia officinalis*) naturally produce this interesting polyphenol compound through oxidating carnosic acid. Furthermore, previous reports have indicated that carnosol has several valuable properties including anti-oxidant, anti-microbial, anti-diabetic, anti-cancer, and immunomodulatory effects [18,19] and modulating peripheral pain signaling [20]. In addition, ample evidence has indicated carnosol stimulates and increases levels of nuclear factor erythroid-derived 2-related factor 2 (Nrf2) displaced into the nucleus [21, 22].

Based on the current and relevant literature, we aimed to appraise the influences of carnosol against LPS-induced inflammation in H9c2 cardiomyoblast and contextually analyze protein and gene levels related to TNF-*α*, IL-1*β*, IL-6, and COX-2. Furthermore, the potential modulation of the NF-*κ*B pathway was investigated using *in silico* molecular docking studies.

## 2. Materials and Methods

### 2.1. Reagents and Kits

Fetal bovine serum (FBS), Griess reagent (G4410 SIGMA), Dulbecco's modified eagle's F12 ham medium (DMEM-F12), antibiotics (penicillin/streptomycin and Fungizone®), lipopolysaccharides (LPS), and other cell culture supplies were obtained from Sigma-Aldrich Chemical Co. (St. Louis, MO, USA). The 3-(4,5-dimethylthiazol-2-yl)- 2,5-diphenyl tetrazolium bromide (MTT) dye was purchased from Roche Diagnostic (Mannheim, Germany). Enzyme-linked immunosorbent assay (ELISA) kits consisting of TNF−*α*, prostaglandin *E*_2_ (PGE_2_), IL-1*β*, and IL-6 were bought from eBioscience (San Diego, CA, USA). TriPure Isolation and cDNA synthesis kits were prepared from Roche Applied Science (Mannheim, Germany) and Fermentase (St. Leon-Rot, Germany), respectively. The glutathione (GSH) assay kit was provided by ZellBio Company (GmbH, Germany). All other chemicals and reagents were of analytical grade and were purchased from Sigma-Aldrich Chemical Co. (St. Louis, MO, USA). The H9c2 rat cardiomyoblast cell line was bought from Pasteur Institute, Tehran, Iran.

### 2.2. Cell Culture and Experimental Design

H9c2 rat cardiomyoblast cells were utilized to investigate the protective effects of carnosol (5, 10, and 20 *μ*M) against inflammation resulting through LPS for 24 h, then followed cotreatment with LPS (10 *μ*g/mL) stimulation [23]. H9c2 cells were routinely cultured in RPMI-1640 supplemented with 10% (v/v) FBS and 1% (v/v) penicillin/streptomycin, which was incubated with 5% v/v CO_2_ at 37°C. The effects of carnosol and LPS on cell viability were investigated using the MTT (5 mg/ml) assay. In general, about 7,000 cells were cultured in the 96-well culture plate overnight and then treated with carnosol (5, 10, and 20 *μ*M) for 24 hours and then coincubated with LPS (10 *μ*g/mL) for subsequent further 24 h. Finally, the optical density (OD) absorbance was read at 540 nm with an ELISA plate reader (STATFAX 2100). The second experiment was designed according to the results of the first experiment to explain the anti-inflammatory mechanism of carnosol. In this regard, H9c2 cells were treated with carnosol, BAY 11-7082, as an inhibitor of the NF-*κ*B pathway, or the combination of carnosol and BAY 11-7082 was then coincubated with LPS as same as the experiment one. In the next step, an MTT assay was conducted to evaluate the effect of BAY 11-7082, carnosol, or LPS on cell viability. First, 96 wells containing 7,000 cells/mL were treated with BAY 11-7082 (12.5–25 *μ*M), and then the plate was incubated for 30 minutes. Thereafter, carnosol (10 *μ*M) was added to each well, and the plate was then incubated for 23.5 h at 37°C. After that, LPS (10 *μ*g/ml) was added to the medium and coincubated for another 24 h. The cells' grouping and treatment for experiments one and two are illustrated in Figures 1 and 2, respectively.

### 2.3. Appraisal of Inflammatory Mediators Levels

After the cell treatment in the first and second experiments (at a density of 2 × 10^6^ cell/well), the supernatant of cells was gathered to measure the secretory levels of inflammatory mediators TNF-*α*, IL-1*β*, IL-6, and PGE_2_, according to the manufacturer's protocol with the help of the corresponding ELISA kits [23, 24].

### 2.4. Assessment of Gene Expression by Quantitative PCR (qPCR)

Based on the manuals, the total RNA was extracted from H9c2 (at a density of 2 × 10^6^ cell/well) treated cells by the TriPure Isolation kit. At the next step, 2 *μ*g of purified RNA was also reversely transcripted to cDNA by cDNA synthesis kit based on the manufacturers' guidelines. Then, the real-time PCR was carried out using the SYBR Green master mix, which was described in our previous reports using the 2^−ΔΔCt^, where Ct represents the threshold cycle number [23, 24]. The primers' sequences (from 5′ to 3′) [23–25] were as follows: TNF-*α*, forward: AAATGGGCTCCCTCTCATCAGTTC and reverse: TCTGCTTGGTGGTTTGCTACGAC; COX-2, forward: TGTATGCTACCATCTGGCTTCGG and reverse: GTTTGGAACAGTCGCTCGTCATC; IL-1*β*, forward: CACCTCTCAAGCAGAGCACAG and reverse: GGGTTCCATGGTGAAGTCAAC; IL-6, forward: TCCTACCCCAACTTCCAATGCTC and reverse: TTGGATGGTCTTGGTCCTTAGCC; and glyceraldehyde 3-phosphate dehydrogenase (GAPDH), forward: GTATTGGGCGCCTGGTCACC and reverse: CGCTCCTGGAAGATGGTGATGG. The GAPDH gene was the reference gene to normalize the expression data.

### 2.5. Statistical Data Analysis

All collected information is displayed as means ± standard deviation (SD) and was analyzed using GraphPad Prism 8.0 software (San Diego, CA, USA) and one-way analysis of variance (ANOVA) and then with Tukey's multiple comparisons tests. Eventually, when *P* < 0.05 was reached, data were considered statistically significant.

### 2.6. Input Files Preparation and Molecular Docking

Docking investigations were carried out using the crystal form of molecular targets NF-kBp65 (1NFI) [26] and IKK [27]. Furthermore, the Schrödinger Protein Preparation Wizard workflow (Schrödinger Suite 2017-1: Protein Preparation Wizard, Schrödinger, LLC, New York, NY, 2021) was considered for preparing the Protein 3D input file from the X-ray structures in the Protein DataBank (PDB) database. Imprimis, water molecules were omitted, and the end of the caps was enclosed. All hydrogen atoms were subjoined in the next step, and bond orders were authorized. In conclusion, the PDB results were formatted in the Maestro (.mae) files. Thereafter, with the help of Maestro's Build Panel (Maestro, Schrödinger, LLC, New York, NY, 2021), the carnosol chemical structure was made and later refined by considering LigPrep software (LigPrep, Schrödinger, LLC, New York, NY, 2021).

For assessing carnosol interactions with IKK*β*, the centroid of the cocrystallized inhibitor [27] ligand was considered as leading to building the necessary molecular docking grid and extending the interior box by 10 Å and the exterior box by 20 Å in the three-dimensional space.

However, there is no NF-kBp65 protein crystal structure complex with a ligand in the PDB. Thus, as also reported in our previous work [28], the Site Map algorithm (SiteMap, Schrödinger, LLC, New York, NY, 2021) was applied for identifying the binding sites [28–30], accordingly. As a result, the Site Map algorithm recommended the five most likely binding sites on the NF-kBp65 protein surface, which were then applied in molecular docking experiments.

The Glide software (Glide, Schrödinger, LLC, New York, NY, 2021) was utilized for all *in silico* docking studies [31–33]. In the beginning, for expanding the sampling mode, 10,000 ligand poses were considered for the initial phase of docking, which was refined to 800 ligand poses by energy minimization. Experimentally, one resulting structure that fulfilled the following parameters, including van der Waals radii = 0.8 and relative charge cutoff = 0.15, was preserved for every ligand. Then, the postdocking optimization of the docking poses was carried out, attributing for an utmost of 50 poses according to a 0.5 kcal/mol refusal limit for the reached at least poses, then submitted for the visual inspection.

## 3. Results

### 3.1. The Impacts of Carnosol on Cell Viability

Our results indicated that incubation with carnosol alone for 48 h provided no cytotoxicity impacts on the H9c2 cells (Figure 3(a)). However, cell viability was meaningfully reduced in the presence of LPS (*P* < 0.001 vs. control; Figure 3(b)). Conversely, different concentrations of carnosol (5, 10, and 20 *μ*M) significantly and concentration-dependently prevented the cell viability reduction against LPS-induced toxicity (*P* < 0.001–0.05; Figure 3(b)).

### 3.2. The Impacts of Carnosol on Inflammatory Biomarkers Levels

The impacts of carnosol and LPS on the gene expression (Figure 4) and protein (Figure 5) levels of inflammatory biomarkers TNF-*α*, IL-1*β*, IL-6, PGE_2_, and COX-2 were examined. LPS significantly upregulated both the gene expression protein levels of TNF-*α* (*P* < 0.001; Figures 4(a) and 5(a)), IL-1*β* (*P* < 0.001; Figures 4(b) and 5(b)), IL-6 (*P* < 0.001; Figures 4(c) and 5(c)), and COX-2 (*P* < 0.001; Figures 4(d) and 5(d)) compared to the control group. On the contrary, pretreatment with carnosol (5, 10, and 20 *μ*M) led to a notable reduction in the gene expression levels of TNF-*α* (*P* < 0.001 vs. LPS for all concentrations; Figure 4(a)), IL-1*β* (*P* < 0.001 vs. LPS for all concentrations; Figure 4(b)), IL-6 (*P* < 0.001 vs. LPS for all concentrations; Figure 4(c)), and COX-2 (*P* < 0.001 vs. LPS for all concentrations; Figure 4(d)) in a concentration-dependent manner. Our results also showed that the treatment of cells with two higher concentrations of carnosol (10 and 20 *μ*M) notably reduced the levels of TNF-*α* (*P* < 0.001 vs. LPS for both cases; Figure 5(a)), IL-1*β* (*P* < 0.001 vs. LPS for both cases; Figure 5(b)), IL-6 (*P* < 0.001 vs. LPS for both cases; Figure 5(c)), and PGE_2_ (*P* < 0.001 vs. LPS for both cases; Figure 5(d)). However, carnosol at the lowest concentration (5 *μ*M) significantly attenuated the levels of TNF-*α* (*P* < 0.001; Figure 5(a)), IL-1*β* (*P* < 0.001; Figure 5(b)), and IL-6 (*P* < 0.01; Figure 5(c)) in comparison to the LPS group.

### 3.3. The Combined Impacts of Carnosol and BAY 11-7082 on LPS-Induced Cytotoxicity

The effects of BAY 11-7082 (12.5 and 25 *μ*M), carnosol (10 *μ*M), and their combination were evaluated on cell viability in the presence and absence of LPS (10 *μ*g/ml) exposure. As shown in Figure 6(a), no significant difference was seen in the cells treated with carnosol (10 *μ*M) and BAY 11-7082 (12.5 and 25 *μ*M) and their combination compared to the control group. However, BAY 11-7082 (12.5 and 25 *μ*M), carnosol (10 *μ*M), and their combinations significantly propagated the level of cell viability against LPS (10 *μ*g/ml) induced cytotoxicity (*P* < 0.001–0.01; Figure 6(b)).

In addition, the effects of carnosol, BAY 11-7082, and their combinations on the expression and secretory levels of inflammatory mediators TNF-*α*, IL-1*β*, IL-6, and COX-2 were also evaluated on LPS-induced cytotoxicity and inflammation in H9c2 cells (Figures 7and 8). LPS significantly increased the expression and secretory levels of TNF-*α* (*P* < 0.001; Figure 7(a) and 8(a)), IL-1*β* (*P* < 0.001; Figures 7(b) and 8(b)), and IL-6 (*P* < 0.001; Figure 7(c) and 8(c)) as well as COX*-*2 (*P* < 0.001; Figure 7(d) and 8(d)) compared to the control group. On the contrary, pretreatment of the cells with BAY 11-7082 (12.5 *μ*M) and carnosol (10 *μ*M) and their combination significantly ameliorated the gene expression levels of TNF-*α* (*P* < 0.001 vs. LPS for all cases; Figure 7(a)), IL-1*β* (*P* < 0.001 vs. LPS for all cases; Figure 7(b)), and IL-6 (*P* < 0.001 vs. LPS for all cases; Figure 7(c)) as well as COX-2 (*P* < 0.001 vs. LPS for all cases; Figure 7(d)) in comparison to the LPS group. Our findings also indicated that pretreatment of the cells with carnosol (10 *μ*M) and BAY 11-7082 (12.5 *μ*M) and their combination significantly diminished the levels of TNF-*α* (*P* < 0.001 vs. LPS for all cases; Figure 8(a)), IL-1*β* (*P* < 0.001 vs. LPS for all cases; Figure 8(b)), and IL-6 (*P* < 0.001 vs. LPS for all cases; Figure 8(c)) as well as PGE_2_ (*P* < 0.001 vs. LPS for all cases; Figure 8(d)) in comparison to the LPS group.

### 3.4. *In Silico* Analysis of Carnosol Interactions with NF-kBp65 and IKK

To propose a binding mode of carnosol with the catalytic domain of IKK*β*, we used the crystal structure of this kinase in a complex with an inhibitor (PDB code: 3RZF), which was applied for computation of molecular docking poses (Figure 9(a)).

From the structural perspective, carnosol was conveniently incorporated in the binding site, like the known inhibitor, making hydrophobic and polar contacts with the target counterpart, making (^1^H) hydrogen bonds with Asp103 and Glu149 (Figure 9(a)).

Due to no crystal structures containing NF-kBp65 (1NFI) [26] in complex with small molecules, we utilized the Sitemap software to disclose the putative binding sites on the macromolecule surface. From the *in silico* simulation, five best putative binding sites as possible interacting regions were revealed. The best site detected overlaps with the DNA-binding domain between the NFkB and the p65 subunits; thus, it was used as a putative pharmacological site of interest. From the detailed computational analysis of ligand/target complex, the diterpenoid makes -cation interaction with Lys28 and two hydrogen bonds with Arg30 and Glu22 (Figure 9(b)).

Interestingly, Arg30 is a protected and critical residue settled in the domain of the DNA-binding inner part of the RxxRxRxxC motif in the loop L1. Indeed, its methylation comprises the binding with DNA [34–36]. Thus, it could be proposed that interactions with Arg30 could inhibit the methylation process [28] and barricade the interaction between the NF-kBp65 subunit and the DNA activating sites.

## 4. Discussion

The current study aimed to explore the promising beneficial effects of carnosol in LPS-associated cytotoxicity in H9c2 cells. The obtained data showed that cell viability was significantly reduced, while both the gene expression and protein levels of inflammatory mediators, including TNF-*α*, IL-1*β*, IL-6, and COX-2, were markedly increased following the LPS stimulation. Noteworthy, we found that treatment with carnosol (5, 10, and 20 *μ*M) or BAY 11-7082) protected H9c2 cardiomyoblast cells against LPS-induced cytotoxicity and inflammation in a concentration-dependent manner.

Inflammation plays a crucial role in cardiovascular disease development, including hypertension, atherosclerosis, acute ischemia-reperfusion injury, postinfarction myocardial remodeling, and atrial fibrillation [5, 24, 37–39] and several molecular signaling pathways suggested for describing impacts of proinflammatory mediators on cardiovascular diseases [2, 5, 37–39]. In this context, inflammation induced by infection has been proposed to cause myocardial dysfunction [8]. LPS, a potent stimulus of inflammation, by its ligand and binding to TLR-4 in cardiomyocytes, activates inflammatory signaling pathways such as NF-*κ*B, allowing the overexpression and overproduction of inflammatory mediators such as IL-1*β*, IL-6, and TNF-*α*, and finally leads to septic shock [39–41]. Considering the previous studies, we used LPS as proinflammatory stimuli on H9c2 cells to mimic, *in vitro*, the etiology of myocarditis. Following the LPS exposure and the reduction of cell viability, the expression and secretory levels of TNF-*α*, IL-1*β*, IL-6, PGE_2_, and COX-2 were upregulated.

Furthermore, in the present study, we found that pretreatment of the H9c2 cells with various concentrations of carnosol (5, 10, and 20 *μ*M) could significantly prevent the LPS-induced cardiomyocytes dysregulation. In agreement with the current findings, Zheng et al. revealed that the expression of IL-1*β* and TNF-*α*, known as the most significant proinflammatory cytokines, were reduced in the kidney tissues of carnosol-treated rats [42]. Moreover, Shi et al. found that treatment of THP-1 cells, primary macrophages derived from murine bone marrow, and human peripheral blood mononuclear cells with carnosol reduced inflammasome activation [43]. Also, Li et al. reported that the differentiation of Th17 cells, known as a subset of proinflammatory T helper cells, was inhibited by carnosol [44]. In addition, the results of *in vitro* studies revealed that carnosol suppressed TNF-*α*-activated NF-*κ*B signaling in human hepatoma cell line HepG2 [21] and IL-6 expression [19]. Accordingly, Momozane et al. showed that carnosol reduced IL-6 gene expression levels in macrophages treated with LPS [45]. Indeed, the current literature supports the present study's hypothesis and confirms the critical role of carnosol in reducing the proinflammatory cytokines and the following deteriorating effects of inflammation and sepsis.

Successively, we evaluated the role of the NF-*κ*B pathway using related inhibitor BAY 11-7082 during the carnosol protection. The current experiment results demonstrated that a combination of carnosol and an NF-*κ*B inhibitor BAY 11-7082 reduces proinflammatory mediators' expression and secretory levels significantly (TNF-*α*, IL-1*β*, IL-6, and PGE_2_ and COX-2).

NF-*κ*B, as the central mediator of immune and inflammation response pathways, is induced via many stimuli, which link to TNF receptor (TNFR), IL-1 receptor (IL-1R), TLRs, and antigen receptors [46–49]. In the cytosol of resting cells, NF-*κ*B is sequestered by the inhibitor of *κ*B (I*κ*B) molecules, preventing the displacement of NF-*κ*B into the nucleus. Thus, the transcriptional function of NF-*κ*B is inhibited and dependent on stimuli [49, 50]. After TNFR, IL-1R, and TLRs activation, the inhibitor of *κ*B kinase (IKK) is activated in the cytosol and phosphorylated, which degrades I*κ*B molecules. There are many reports regarding BAY 11-7082 as an NF-*κ*B signaling pathway inhibitor and its anti-inflammatory effect. Indeed, in a study conducted by Lee et al., results demonstrated that phosphorylation of p50 and p65 (as subunits of NF-*κ*B) was suppressed by BAY 11-7082 [51]. Juliana et al. have indicated the NLRP3 inflammasome, which is activated via virus and bacteria and induces the production of IL-1*β*, is inhibited by BAY 11-7082 [52]. Moreover, results obtained from research in the rat myocardial ischemia/reperfusion (IR) injury model showed that BAY 11-7082 declined inflammation and apoptosis in myocardial cells and decreased the infarct size [53]. Finally, Irrera et al. showed that BAY 11-7082 reduced the expression of proinflammatory cytokines such as TNF-*α*, IL-1*β*, IL-6, and IL-23 [54]. In our study, we found that BAY 11-7082 had protective effects in a similar way to carnosol, thus speculating that carnosol may exert its anti-inflammatory influence by the NF-*κ*B pathway. On these bases, we have used the *in silico* methodologies to rationalize the structural molecular interactions between carnosol and IKK and NF-*κ*B. Hence, the pattern of hydrogen bonds and the number of hydrophobic contacts both with sites of pharmacological interest domain seem to be the driving forces of the target-ligand complexes. Lo et al. conducted a study on mouse macrophages being treated with carnosol and indicated that the activation of NF-*κ*B was suppressed [55]. Furthermore, another study conducted by Wang et al. demonstrated that carnosol via upregulation of Nrf-2 and downregulation of NF-*κ*B and COX-2 protects against spinal cord injury [56].

The results showed that COX-2 gene expression and PGE_2_ levels in treated cells with carnosol, BAY 11-7082, and the combination of carnosol and BAY 11-7082 were reduced compared to the LPS group. Thus, it seems that COX-2 was strongly stimulated via activating NF-*κ*B in response to LPS in H9C2 cardiomyocytes. As reported by Pang et al., NF-*κ*B is a leading mediator for expressing COX-2 in H9c2 cardiomyoblast [37]. Cyclooxygenase (COX) enzymes aimed to catalyze arachidonic acid conversion to prostaglandins and had two isoforms, COX-1 and COX-2. Opposite to COX-1, known as the housekeeping enzyme, the COX-2 expression was significantly induced in response to different stimuli and regarded as an inducible isoform, while under physiological conditions, it had shallow expression [37, 57, 58]. For instance, COX-2 can be overexpressed through stimulation with LPS [59, 60]. Furthermore, it was proved that the expression of COX-2 in the cardiac cells increased during myocardial ischemia. Thus, it is proposed that such an enzyme can be involved in ischemic heart disease [37].

Furthermore, it was reported that PGE_2_ can be predominantly produced through COX-2 and is responsible for the signs and symptoms of inflammation associated with sepsis [59]. This study proposed that carnosol suppressed the LPS-associated with overexpression of COX-2, causing the attenuation of PGE_2_ secretion. A study performed by Lee et al. indicated that carnosol reduced inflammation and COX-2 expression in skin cells among rats [61]. Furthermore, the results obtained from another study on the rats treated with carnosol indicated that it inhibited COX-2 activity [62].

## 5. Conclusion

In summary, the current study explicit that carnosol had no toxic impacts on H9c2 cells but alleviated LPS-induced cardiomyoblast toxicity. Besides, the promising protective results of carnosol against LPS-induced inflammation in H9c2 cardiomyoblast through inhibiting the NF-*κ*B signaling pathway. Thus, carnosol may have defensive consequences against sepsis-induced myocardial and other inflammatory diseases involving the NF-*κ*B signaling pathway, including myocarditis and inflammatory cardiomyopathy. At the same time, more cellular animal experiments are required for specifying the mechanisms precisely and scaling to the clinics.

## Figures and Tables

**Figure 1:** Grouping the cell line H9c2 and treating with carnosol (CA) and LPS. ^*∗*^Completed media culture without LPS.

**Figure 2:** Grouping the cell line H9c2 and treating with BAY 11-7082, carnosol (CA), and LPS. ^*∗*^Completed media culture without LPS.

**Figure 3:** The impacts of carnosol on the level of cell viability without (a) or with LPS-induced toxicity (b). Data were represented as mean ± SD (*n* = 6); ^###^*P* < 0.001*versus* control; and ^*∗*^*P* < 0.05, ^*∗∗*^*P* < 0.01, and ^*∗∗*^^*∗*^*P* < 0.001*versus* LPS.

**Figure 4:** Effects of carnosol (CA) and LPS on the gene expression levels of (a) TNF-*α*, (b) IL-1*β*, (c) IL-6, and (d) COX-2. The real-time PCR method was applied to assess gene expression levels, and the results were normalized to the control group. The reference gene was GAPDH. Data were displaced as mean ± SD (*n* = 6); ^###^*P* < 0.001*versus* control; and ^*∗∗*^^*∗*^*P* < 0.001*versus* LPS.

**Figure 5:** The effects of carnosol (CA) and LPS on the protein levels of (a) TNF-*α*, (b) IL-1*β*, (c) IL-6, and (d) PGE_2_. The secretory levels of inflammatory mediators were measured using the ELISA method. Data were presented as mean ± SD (*n* = 6); ^###^*P* < 0.001 versus control; and ^*∗∗*^^*∗*^*P* < 0.001 and ^*∗∗*^*P* < 0.01 versus LPS.

**Figure 6:** The impacts of carnosol (CA; 10 *μ*M), BAY 11-7082 (BAY; 12.5 and 25 *μ*M), and their combinations on the levels of cell viability in the absence (a) or presence of LPS-induced toxicity (b). Data were represented as mean ± SD (*n* = 6); ^###^*P* < 0.001*versus* control; and ^*∗∗*^*P* < 0.01 and ^*∗∗*^^*∗*^*P* < 0.001*versus* LPS.

**Figure 7:** The influences of BAY 11-7082 (BAY; 12.5 *μ*M), carnosol (CA; 10 *μ*M), and their combinations on the gene expression levels of (a) TNF-*α*, (b) IL-1*β*, (c) IL-6, and (d) COX-2 against LPS-induced cytotoxicity. The real-time PCR method was applied to assess gene expression levels, and the results were normalized to the control group. The reference gene was GAPDH. Data were illustrated as mean ± SD (*n* = 6); ^###^*P* < 0.001 versus control; and ^*∗∗*^^*∗*^*P* < 0.001 versus LPS.

**Figure 8:** The impacts of BAY 11-7082 (BAY; 12.5 *μ*M), carnosol (CA; 10 *μ*M), and their combinations on the secretory levels of inflammatory mediators: (a) TNF-*α*, (b) IL-1*β*, (c) IL-6, and (d) PGE_2_ against LPS-induced cytotoxicity. The protein levels were assessed using the ELISA technique. Data were illustrated as mean ± SD (*n* = 6); ^###^*P* < 0.001 versus control; and ^*∗∗∗*^*P* < 0.001 versus LPS.

**Figure 9:** 3D-model of the carnosol (yellow sticks) in the binding sites of IKK*β* (reported in green sticks and ribb ons in panel (a)) and NF-kBp65 (reported in cyan sticks and ribbons in panel (b)). Hydrogen bonds are illustrated as yellow dotted lines, and *π*-*π* stacking interactions are designated as green dotted lines. Known inhibitor of IKK*β* is reported as cyan sticks in panel A.

## Data Availability

The data sets used and/or analyzed during the current study are available from the corresponding author on reasonable request.

## Abbreviations

MTT: 3-(4,5-dimethylthiazol-2-yl)-2,5-diphenyl tetrazolium bromide
COX-2: Cyclooxygenase-2
COX: Cyclooxygenase
DMEM-F12: Dulbecco's modified eagle's F12 ham medium
ELISA: Enzyme-linked immunosorbent assay
FBS: Fetal bovine serum
GSH: Glutathione
GAPDH: Glyceraldehyde 3-phosphate dehydrogenase
IL-1R: IL-1 receptor
IL-1*β*: Interleukin
LPS: Lipopolysaccharide
NF-*κ*B: Nuclear factor-kappa B
ANOVA: One-way analysis of variance
PDB: Protein DataBank
qPCR: Quantitative PCR
TNFR: TNF receptor
TLR-4: Toll-like receptor-4
TNF-*α*: Tumor necrosis factor
VEGF: Vascular endothelial growth factor.

## References

[1] Ghasemian M., Owlia S., Owlia M. B. (2016). Review of anti-inflammatory herbal medicines. *Advances in pharmacological sciences*.

[2] Rahimi V. B., Askari V. R., Shirazinia R. (2018). Protective effects of hydro-ethanolic extract of Terminalia chebula on primary microglia cells and their polarization (M1/M2 balance). *Multiple Sclerosis and Related Disorders*.

[3] Ye H., Wang Y., Jenson A. B., Yan J. (2016). Identification of inflammatory factor TNF*α* inhibitor from medicinal herbs. *Experimental and Molecular Pathology*.

[4] Yim M.-J., Lee J. M., Choi G. (2018). Anti-inflammatory potential of carpomitra costata ethanolic extracts via inhibition of nf-*κ*B and ap-1 activation in lps-stimulated raw264. 7 macrophages. *Evidence-Based Complementary and Alternative Medicine*.

[5] Baradaran Rahimi V., Rajabian A., Rajabi H. (2020). The effects of hydro-ethanolic extract of Capparis spinosa (C. spinosa) on lipopolysaccharide (LPS)-induced inflammation and cognitive impairment: evidence from in vivo and in vitro studies. *Journal of Ethnopharmacology*.

[6] Drosatos K., Lymperopoulos A., Kennel P. J., Pollak N., Schulze P. C., Goldberg I. J. (2015). Pathophysiology of sepsis-related cardiac dysfunction: driven by inflammation, energy mismanagement, or both?. *Current Heart Failure Reports*.

[7] Franceschelli S., Pesce M., Ferrone A. (2017). Biological effect of licochalcone C on the regulation of PI3K/Akt/eNOS and NF-*κ*B/iNOS/NO signaling pathways in H9c2 cells in response to LPS stimulation. *International Journal of Molecular Sciences*.

[8] Luo Q., Yang A., Cao Q., Guan H. (2018). 3, 3′-Diindolylmethane protects cardiomyocytes from LPS-induced inflammatory response and apoptosis. *BMC Pharmacology and Toxicology*.

[9] Askari V. R., Baradaran Rahimi V., Assaran A., Iranshahi M., Boskabady M. H. (2019). Evaluation of the anti-oxidant and anti-inflammatory effects of the methanolic extract of Ferula szowitsiana root on PHA-induced inflammation in human lymphocytes. *Drug and Chemical Toxicology*.

[10] Liu L., Liu F., Sun Z., Peng Z., You T., Yu Z. (2020). LncRNA NEAT1 promotes apoptosis and inflammation in LPS-induced sepsis models by targeting miR-590-3p. *Experimental and Therapeutic Medicine*.

[11] Martins G. R., Gelaleti G. B., Moschetta M. G., Maschio-Signorini L. B., Zuccari D. A., De Campos P. (2016). Pro-inflammatory and Anti-inflammatory Cytokines Mediated by NF-*κ*B Factor as Prognostic Markers in Mammary Tumors. *Mediators of inflammation*.

[12] Askari V. R., Baradaran Rahimi V., Tabatabaee S. A., Shafiee-Nick R. (2019). Combination of Imipramine, a sphingomyelinase inhibitor, and *β*-caryophyllene improve their therapeutic effects on experimental autoimmune encephalomyelitis (EAE). *International Immunopharmacology*.

[13] Yahfoufi N., Alsadi N., Jambi M., Matar C. (2018). The immunomodulatory and anti-inflammatory role of polyphenols. *Nutrients*.

[14] Ko S.-G., Yin C. S., Du B., Kim K. (2014). Herbal medicines for inflammatory diseases. *Mediators of Inflammation*.

[15] Schwager J., Richard N., Fowler A., Seifert N., Raederstorff D. (2016). Carnosol and related substances modulate chemokine and cytokine production in macrophages and chondrocytes. *Molecules*.

[16] Mena P., Cirlini M., Tassotti M., Herrlinger K. A., Dall’Asta C., Del Rio D. (2016). Phytochemical profiling of flavonoids, phenolic acids, terpenoids, and volatile fraction of a rosemary (Rosmarinus officinalis L.) extract. *Molecules*.

[17] Roohbakhsh Y., Baradaran Rahimi V., Silakhori S. (2020). Evaluation of the effects of peritoneal lavage with rosmarinus officinalis extract against the prevention of postsurgical-induced peritoneal adhesion. *Planta Medica*.

[18] Yan M., Vemu B., Veenstra J., Petiwala S. M., Johnson J. J. (2018). Carnosol, a dietary diterpene from rosemary (Rosmarinus officinalis) activates Nrf2 leading to sestrin 2 induction in colon cells. *Integrative molecular medicine*.

[19] Sanchez C., Horcajada M.-N., Scalfo F. M., Ameye L., Offord E., Henrotin Y. (2015). Carnosol inhibits pro-inflammatory and catabolic mediators of cartilage breakdown in human osteoarthritic chondrocytes and mediates cross-talk between subchondral bone osteoblasts and chondrocytes. *PLoS One*.

[20] Maione F., Cantone V., Pace S. (2017). Anti-inflammatory and analgesic activity of carnosol and carnosic acid in vivo and in vitro and in silico analysis of their target interactions. *British Journal Pharmacol*.

[21] Chen C.-C., Chen H.-L., Hsieh C.-W., Yang Y.-L., Wung B.-S. (2011). Upregulation of NF-E2-related factor-2-dependent glutathione by carnosol provokes a cytoprotective response and enhances cell survival. *Acta Pharmacologica Sinica*.

[22] O’Neill E. J., Den Hartogh D. J., Azizi K., Tsiani E. (2020). Anticancer properties of carnosol: a summary of in vitro and in vivo evidence. *Antioxidants (Basel)*.

[23] Taherzadeh D., Baradaran Rahimi V., Amiri H. (2022). Acetyl-11-Keto-*β*-Boswellic acid (AKBA) prevents lipopolysaccharide-induced inflammation and cytotoxicity on H9C2 cells. *Evidence-based Complementary and Alternative Medicine*.

[24] Rahim V. B., Khammar M. T., Rakhshandeh H., Samzadeh-Kermani A., Hosseini A., Askari V. R. (2019). Crocin protects cardiomyocytes against LPS-Induced inflammation. *Pharmacological Reports*.

[25] Peinnequin A., Mouret C., Birot O. (2004). Rat pro-inflammatory cytokine and cytokine related mRNA quantification by real-time polymerase chain reaction using SYBR green. *BMC Immunology*.

[26] Jacobs M. D., Harrison S. C. (1998). Structure of an I*κ*B*α*/NF-*κ*B complex. *Cell*.

[27] Xu G., Lo Y.-C., Li Q. (2011). Crystal structure of inhibitor of *κ*B kinase *β*. *Nature*.

[28] Maione F., Piccolo M., De Vita S. (2018). Down regulation of pro-inflammatory pathways by tanshinone IIA and cryptotanshinone in a non-genetic mouse model of Alzheimer’s disease. *Pharmacological Research*.

[29] Halgren T. (2007). New method for fast and accurate binding-site identification and analysis. *Chemical Biology & Drug Design*.

[30] Halgren T. A. (2009). Identifying and characterizing binding sites and assessing druggability. *Journal of Chemical Information and Modeling*.

[31] Friesner R. A., Banks J. L., Murphy R. B. (2004). Glide: a new approach for rapid, accurate docking and scoring. 1. Method and assessment of docking accuracy. *Journal of Medicinal Chemistry*.

[32] Friesner R. A., Murphy R. B., Repasky M. P. (2006). Extra precision Glide: docking and scoring incorporating a model of hydrophobic enclosure for Protein−Ligand complexes. *Journal of Medicinal Chemistry*.

[33] Halgren T. A., Murphy R. B., Friesner R. A. (2004). Glide: a new approach for rapid, accurate docking and scoring. 2. Enrichment factors in database screening. *Journal of Medicinal Chemistry*.

[34] Harris D. P., Bandyopadhyay S., Maxwell T. J., Willard B., Dicorleto P. E. (2014). Tumor necrosis factor (TNF)-*α* induction of CXCL10 in endothelial cells requires protein arginine methyltransferase 5 (PRMT5)-mediated nuclear factor (NF)-*κ*B p65 methylation. *Journal of Biological Chemistry*.

[35] Reintjes A., Fuchs J. E., Kremser L. (2016). Asymmetric arginine dimethylation of RelA provides a repressive mark to modulate TNF*α*/NF-*κ*B response. *Proceedings of the National Academy of Sciences*.

[36] Wei H., Wang B., Miyagi M. (2013). PRMT5 dimethylates R30 of the p65 subunit to activate NF- B. *Proceedings of the National Academy of Sciences*.

[37] Pang L., Cai Y., Tang E. H. C. (2016). Cox-2 inhibition protects against hypoxia/reoxygenation-induced cardiomyocyte apoptosis via Akt-dependent enhancement of iNOS expression. *Oxidative Medicine and Cellular Longevity*.

[38] Tian Y., Song H., Qin W. (2020). Mammalian STE20-like kinase 2 promotes lipopolysaccharides-mediated cardiomyocyte inflammation and apoptosis by enhancing mitochondrial fission. *Frontiers in Physiology*.

[39] Zhang X., Zhao Y., Bai D., Yuan X., Cong S. (2019). Schizandrin protects H9c2 cells against lipopolysaccharide‐induced injury by downregulating Smad3. *Journal of Biochemical and Molecular Toxicology*.

[40] Curtis M. J., Bond R. A., Spina D. (2015). Experimental design and analysis and their reporting: new guidance for publication in BJP. *British Journal of Pharmacology*.

[41] Hao R., Su G., Sun X., Kong X., Zhu C., Su G. (2019). Adiponectin attenuates lipopolysaccharide-induced cell injury of H9c2 cells by regulating AMPK pathway. *Acta Biochimica et Biophysica Sinica*.

[42] Zheng Y., Zhang Y., Zheng Y., Zhang N. (2018). Carnosol protects against renal ischemia-reperfusion injury in rats. *Experimental Animals*.

[43] Shi W., Xu G., Zhan X. (2020). Carnosol inhibits inflammasome activation by directly targeting HSP90 to treat inflammasome-mediated diseases. *Cell Death & Disease*.

[44] Li X., Zhao L., Han J.-J. (2018). Carnosol modulates Th17 cell differentiation and microglial switch in experimental autoimmune encephalomyelitis. *Frontiers in Immunology*.

[45] Momozane T., Kawamura T., Itoh Y. (2018). Carnosol suppresses interleukin-6 production in mouse lungs injured by ischemia–reperfusion operation and in RAW264. 7 macrophages treated with lipopolysaccharide. *Biochemistry and Cell Biology*.

[46] Abraham E. (2003). Nuclear factor-*κ*B and its role in sepsis‐associated organ failure. *The Journal of Infectious Diseases*.

[47] Armistead B., Kadam L., Drewlo S., Kohan-Ghadr H.-R. (2020). The role of NF*κ*B in healthy and preeclamptic placenta: trophoblasts in the spotlight. *International Journal of Molecular Sciences*.

[48] Hoesel B., Schmid J. A. (2013). The complexity of NF-*κ*B signaling in inflammation and cancer. *Molecular Cancer*.

[49] Mussbacher M., Salzmann M., Brostjan C. (2019). Cell type-specific roles of NF-*κ*B linking inflammation and thrombosis. *Frontiers in Immunology*.

[50] Baker R. G., Hayden M. S., Ghosh S. (2011). NF-*κ*B, inflammation, and metabolic disease. *Cell Metabolism*.

[51] Lee J., Rhee M. H., Kim E., Cho J. Y. (2012). BAY 11-7082 is a broad-spectrum inhibitor with anti-inflammatory activity against multiple targets. *Mediators of inflammation*.

[52] Juliana C., Fernandes-Alnemri T., Wu J. (2010). Anti-inflammatory compounds parthenolide and Bay 11-7082 are direct inhibitors of the inflammasome. *Journal of Biological Chemistry*.

[53] Kim Y. S., Kim J. S., Kwon J. S. (2010). BAY 11-7082, a nuclear factor-*κ*B inhibitor, reduces inflammation and apoptosis in a rat cardiac ischemia-reperfusion injury model. *International Heart Journal*.

[54] Irrera N., Vaccaro M., Bitto A. (2017). BAY 11-7082 inhibits the NF-*κ*B and NLRP3 inflammasome pathways and protects against IMQ-induced psoriasis. *Clinical Science*.

[55] Lo A.-H., Liang Y.-C., Lin-Shiau S.-Y., Ho C.-T., Lin J.-K. (2002). Carnosol, an antioxidant in rosemary, suppresses inducible nitric oxide synthase through down-regulating nuclear factor-*κ*B in mouse macrophages. *Carcinogenesis*.

[56] Wang Z.-H., Xie Y.-X., Zhang J.-W. (2016). Carnosol protects against spinal cord injury through Nrf-2 upregulation. *Journal of Receptors and Signal Transduction*.

[57] Attiq A., Jalil J., Husain K., Ahmad W. (2018). Raging the war against inflammation with natural products. *Frontiers in Pharmacology*.

[58] Martín-Sanz P., Hortelano S., Boscá L., Casado M. (2006). Cyclooxygenase 2: understanding the pathophysiological role through genetically altered mouse models. *Frontiers in Bioscience*.

[59] Lin C.-Y., Wang W.-H., Chen S.-H. (2017). Lipopolysaccharide-induced nitric oxide, prostaglandin E2, and cytokine production of mouse and human macrophages are suppressed by pheophytin-b. *International Journal of Molecular Sciences*.

[60] Lin C. H., Lin C. C. (2016). Sitagliptin attenuates inﬂammatory responses in lipopolysaccharide-stimulated cardiomyocytes via nuclear factor-*κ*B pathway inhibition. *Experimental and Therapeutic Medicine*.

[61] Lee D. Y., Hwang C. J., Choi J. Y. (2017). Inhibitory effect of carnosol on phthalic anhydride-induced atopic dermatitis via inhibition of STAT3. *Biomolecules & Therapeutics*.

[62] Emami F., Ali-Beig H., Farahbakhsh S. (2013). Hydroalcoholic extract of Rosemary (Rosmarinus officinalis L.) and its constituent carnosol inhibit formalin-induced pain and inflammation in mice. *Pakistan Journal of Biological Sciences: PJBS*.

